RETRACTED

# Tumor microenvironment and immune system preservation in early-stage breast cancer: routes for early recurrence after mastectomy and treatment for lobular and ductal forms of disease

**DOI:** 10.1186/s12865-023-00591-y

**Published:** 2024-01-25

**Authors:** Hassan A. Saad, Azza Baz, Mohamed Riad, Mohamed E. Eraky, Ahmed El-Taher, Mohamed I. Farid, Khaled Sharaf, Huda E. M. Said, Lotfy A. Ibrahim

**Affiliations:** 1 Surgical Department, Faculty of Medicine, Zagazig University, Zagazig City, 44661 Egypt; 2 Surgical Department, Alahrar Teaching Hospital, Zagazig University, Zagazig City, 55971 Egypt; 3 Clinical Pathology Department, Faculty of Medicine, Zagazig University, Zagazig City, 55971 Egypt; 4 Surgical Department, AlAzhar University, Nasr City, Cairo 55888 Egypt

**Keywords:** Early breast cancer prediction, Immune microenvironment, Role of immune system in IDC, DCI and ILC

## Abstract

**Background:**

Intra-ductal cancer (IDC) is the most common type of breast cancer, with intra-lobular cancer (ILC) coming in second. Surgery is the primary treatment for early stage breast cancer. There are now irrefutable data demonstrating that the immune context of breast tumors can influence growth and metastasis. Adjuvant chemotherapy may be administered in patients who are at a high risk of recurrence. Our goal was to identify the processes underlying both types of early local recurrences.

**Methods:**

This was a case-control observational study. Within 2 years of receiving adjuvant taxan and anthracycline-based chemotherapy, as well as modified radical mastectomy (MRM), early stage IDC and ILC recurred. Vimentin, α-smooth muscle actin (SMA), platelet-derived growth factor (PDGF), matrix metalloproteinase (MMP1), and clustered differentiation (CD95) were investigated.

**Results:**

Of the samples in the ductal type group, 25 showed local recurrence, and 25 did not. Six individuals in the lobular-type group did not experience recurrence, whereas seven did. Vimentin (*p* = 0.000 and 0.021), PDGF (*p* = 0.000 and 0.002), and CD95 (*p* = 0.000 and 0.045) expressions were significantly different in ductal and lobular carcinoma types, respectively. Measurement of ductal type was the sole significant difference found in MMP1 (*p* = 0.000) and α-SMA (*p* = 0.000). α-SMA and CD95 were two variables that helped the recurrence mechanism in the ductal type according to the pathway analysis. In contrast, the CD95 route is a recurrent mechanism for the lobular form.

**Conclusions:**

While the immune system plays a larger role in ILC, the tumor microenvironment and immune system both influence the recurrence of IDC. According to this study, improving the immune system may be a viable cancer treatment option.

RETRACTED

## Introduction

Breast cancer metastases occur when cancer cells are able to move and endure the body’s defense. These cancer cells must be able to alter the extracellular matrix and cytoskeleton structure to facilitate migration and prevent apoptosis. Innate immunity comprises the initial immune response, occurring within hours of encountering a foreign antigen, and is antigen-independent (non-specific). On the other hand, adaptive immunity is antigen-dependent and pathogen-specific but requires approximately 4–7 days to mount a fully active response. It is well accepted that the immune system has an integral role in shaping the evolution of cancer through the process of immunoediting. As a result, immunotherapy is now part of some cancer treatments, rallying the body’s immune system to fight cancer. Checkpoint inhibitors, for example, have been developed to target and block the immune checkpoint proteins CTLA-4, PD-1, and PD-L1, which are upregulated in tumor and immune cells and restrict the immune system from attacking the tumor. They can accomplish this by creating proteins for self-defense and modifying signaling pathways to prevent apoptosis.

Egypt’s incidence rate is lower than the worldwide average, but its age-standardized death rate—20.4/100,0004—is greater than the rates in the US (12.3/105) and affluent nations (12.8/105) [1–4]. The main cause of these differences in incidence and death between Egypt and other nations has been  identified as the delayed diagnosis presentation. Instead of being in the early stages, the majority of cases in  Egypt present as locally progressed or metastatic [5–8].

Interestingly, this mortality rate is far greater than that of China and other emerging nations, where the agestandardized mortality rate is 6.3/105 [6].

The main cause of these differences in incidence and death between Egypt and other nations has been identified as  the delayed diagnosis presentation. Instead of being in the early stages, the majority of cases in Egypt present as locally progressed or metastatic [4, 7, 8]. There is ongoing debate over which type has a better prognosis. Local recurrence and distant metastases after surgery are more common in patients with ILC. 6 The high number of metastases in ILC is due to the nature of the tumor, which tends to be multicentric and can invade the stroma  without inducing excessive stromal reactions [7, 8].

Breast conserving surgery (BCS) and modified radical mastectomy (MRM) are two common surgical procedures for breast cancer [6, 7]. MRM involves removal of the entire breast, including all the breast glands and skin surrounding the tumor, along with simultaneous axillary dissection [8]. Following MRM, metastases and recurrences are common, even after adjuvant chemotherapy, even though the entire breast has been removed.

RETRACTED

The first 2 years following primary surgery are the most critical periods for local recurrence in both histological types [9, 10]. Re-excision or salvage mastectomy is the option for managing local recurrence following a BCS procedure; however, owing to the high rate of post-re-excision metastases, the choice of procedure is still under debate [11]. Up until date, there has not been a standard approach for managing local recurrence following MRM, such as whether re-excision can be performed or treated in a stage IV environment [9, 12].

Treatment of breast cancer that has metastasized can also result in a reduction in the distant anti-angiogenic effect, which can lead to the formation of new metastatic foci in distant organs [13, 14]. Surgery and chemotherapy can also increase the formation of reactive oxygen species (ROS), which can protect cancer cells from apoptosis through the “anti-ROS” mechanism of Nuclear Factor Kappa Beta (NF-kB). Tumor cells may be shed into the bloodstream and lymph nodes as a result of these procedures. Furthermore, through the Twist signaling pathway, low ROS levels can transform cancer cells into cancer stem cells (CSC) [15].

Cancer cells have the ability to change their nature in order to become immortal (stemness), as well as the ability to invade and migrate in order to live and spread. Cancer cells undergo a transition from an epithelial to a more mobile mesenchymal phenotype via the epithelial-to-mesenchymal transition (EMT) mechanism [16]. One of the mechanisms that renders cancer stem cells (CSCs) immortal is their resistance to immune system-triggered apoptosis, which they avoid by upregulating the expression of CD95, a protein that both triggers and activates [17].

Higher levels of mesenchymal markers such as vimentin, N-cadherin, and fibronectin indicate that cancer cells are undergoing EMT. Epithelial markers, including claudin, E-cadherin, and cytokeratin, were also less expressed [18, 19]. Cancer cells that have undergone EMT have the ability to migrate and spread through a mechanism that can transform normal fibroblast cells into cancer-associated fibroblasts (CAF) via the platelet-derived growth factor (PDGF) pathway [20]. CAF modifies the morphology and structure of fibroblasts to enhance metastatic processes. Increased expression of α-SMA, which is correlated with EMT, can be used to identify CAF formation. Additionally, CAF can send out signals to induce the formation of matrix metalloproteinases (MMP), which degrade the extracellular matrix and facilitate the migration of cancer cells. There are more than 21 different varieties of MMPs and MMP1.29, the expression of which increases in breast cancer. MMP is a proteolytic enzyme that controls the cellular microenvironment.

RETRACTED

## Methods

The present study aimed to elucidate the variations in the local recurrence mechanisms of ductal and lobular invasive breast cancer following mastectomy and chemotherapy. There were two types of breast cancer in this study, and the expression of vimentin, α-SMA, MMP1, PDGF, and CD95 was compared to determine which parts are more important for local recurrence.

approval and agreement to participate in ethics.

The Research Ethics Committee. The data collected from 3 specialised hospital.

### Data techniques

An analytical observational study with a case-control study design was the research design that was employed. During the 5 years from January 2016 to December 2020 (the study period), patients with early stage IDC and ILC (stages I and II) underwent MRM, received chemotherapy using a taxane and anthracycline-based regimen, and experienced local recurrence within 2 years following surgery. The first author performed all the operations. Data were acquired from the medical records of the surgical department by Professor H. A. Saad of General Hospital located in (ZGH) (corresponding author).

### Sampling and patients choice

For each category, the research participants were split into two groups: those with local recurrence and those without. For IDC, there were 25 samples per group. The sample size was calculated based on the minimum of the samples required for regression analysis. Simple random sampling was used as the sampling method for each ductal group. The total number of participants who met the inclusion and exclusion criteria was the number of samples for ILC. This study was conducted in ZGH. The admission and exclusion criteria were as follows:

#### Criteria of inclusion

- 1- As an A. Patients who have undergone six rounds of chemotherapy for taxan and anthracycline base at three-week intervals and who have locoregional recurrence following MRM due to early-stage lobular and ductal invasive breast cancer (one series)
  - Type histological
  - Algebra
  - Adversity
- 2- A report from the anatomic pathology evaluation contained the following:
- 3- The patient’s whole medical history was available, containing the following: 
  - Patient names and ages
  - Hormonal condition of patient

Metastases in local lymph nodes

Surgical date and recurrence time.

- Regimen timing and type of chemotherapy

#### Criteria for exclusion

1. As an A. The patient was not new to radiation treatment.
2. A. Malignancy was present in additional organs.
3. The pathological examination’s findings indicated that the resection’s boundaries were not less than 1 cm, coincident, or tumor-free.

RETRACTED

Day. Because of its deterioration, the paraffin block was not usable.

e. Immunohistochemistry could not examine paraffin blocks from surgical specimens due to inadequate fixing.

After cutting to a thickness of 4 μm, the paraffin block from the MRM operation specimen was heated for an hour at 600 °C. Next, xylene solution was used three times for 3 minutes each time to perform deparaffinization. In addition, ethanol concentrations of 100, 96, and 70% were used for rehydration. Rehydrate, and then give yourself a three-minute water wash. 0.5% H2O2 was used to stop peroxidase activity for 30 min in methanol, followed by washing with water for 5 min. Prior to and following peroxidase blockage, phosphate-buffered saline (PBS) with a pH of 7.4 was used for washing. Mouse Anti-Human Monoclonal Antibody from MyBioSource was used in this investigation. The specific medications used were MBS475544 (vimentin), MBS2507725 (PDGF), MBS476188 (MMP1), MBS266274 (α-SMA), and MBS10754069 (CD95). The antibodies were diluted in phosphate-buffered saline containing bovine serum albumin, optimized at a concentration of 1:600, and incubated for 30 min at room temperature. To evaluate and analyze the collected slides, the number of cells that demonstrated a positive reaction to each antibody was counted. A 400x magnification light microscope was used in this study. Ten fields of view were used for the calculation, and the average number of positive cells in each field of view was calculated. To determine the differences between the group that had a recurrence and the group that did not, statistical analysis was performed.

The mean difference test was used in this study. Homogeneity and normality tests are commonly performed first, followed by a logistic regression test before proceeding with the pathway analysis. OpenEpi version 3.0, which is the data processing software used, and EZR, a free statistical application based on the R-command, were also used. Statistical significance was set at *p* < 0.05.

## Results

### Examine the attributes

Thirteen patients with lobular breast cancer and 50 with early stage ductal breast cancer were included in the study. The ductal type was divided into two groups:25 patients in the first group experienced local recurrence within the first 2 years, whereas the remaining 25 patients in the control group did not experience local recurrence. Within the lobular type group, the number of patients with local recurrence (seven patients) and those without local recurrence (six patients) were likewise divided (Tables 1 and 2).

RETRACTED

**Table 1:** Characteristics of the research sample on the ductal type

Negative recurrence (*n* = 25)	Positive recurrence (*n* = 25)	*p*	
**Age (mean)**	51.72	49.96	0.59
**Lymph node metastases**	3.04	3.92	0.527
**Grade**	1.96	2	0.166
**Hormonal status**			
Pre-menopause	12	14	0.5713
Menopause	13	11

**Table 2:** Characteristics of the research sample on the lobular type

Negative recurrence (*n* = 6)	Positive recurrence (*n* = 7)	*p*	
**Age (mean)**	46.83	51.00	0.532
**Lymph nodes metastases**	1.33	3.00	0.07
**Grade**	1.86	2	0.631
**Hormonal status**			
Pre-menopause	3	5	0.428
Menopause	3	2	

#### Analysis of the data

We checked the data distribution for homogeneity and normality before performing the statistical tests. A parametric independent t-test was employed for data with a normal distribution, whereas a non-parametric Mann-Whitney test was used for data that were not normally distributed.

Table 3 indicates that there was a significant difference in vimentin expression between the recurrence-affected and control groups (*p* = 0.000 for the ductal type and *p* = 0.021 for the lobular type).

**Table 3:** Statistical test results of vimentin expression for ductal and lobular types

Invasive breast cancer type	Vimentin expression		*p*
	Non-recurrence	Recurrence	
Ductal	2.24 ± 1.72	8.32 ± 5.74	0.000*
	1.50 (0.4–7.2)	6.00 (2.3–21.0)	
Lobular	1.43 ± 1.50	8.16 ± 5.75	0.021**
	0.90 (0.0–4.0)	9.10 (1.9–18.5)	
p	0.168*	0.909*	

The Mann-Whitney test *

** Separate t-test

Table 3 Vimentin expression test findings for ductal and lobular types, as determined statistically.

According to the test results, there was a significant difference in PDGF expression in both forms of breast cancer, with *p* = 0.000 for the ductal type and *p* = 0.002 for the lobular type, between the groups that experienced recurrence and those that did not (Table 4).

**Table 4:** Statistical test results of platelet-derived growth factor (PDGF) expression for ductal and lobular types

Invasive breast cancer type	PDGF expression		*p*
	Non-recurrence	Recurrence	
Ductal	3.95 ± 2.70	14.95 ± 5.36	0.000*
	3.20 (0.9–10.7)	15.60 (6.4–24.2)	
Lobular	1.62 ± 1.58	6.96 ± 3.01	0.002**
	1.35 (0.0–4.4)	6.40 (4.0–11.3)	
p	0.030*	0.001**	

The Mann-Whitney test *

** Separate t-test

Table 4 results of a statistical test measuring the expression of platelet-derived growth factor (PDGF) in ductal and lobular types.

The results of the tests showed that in the ductal type group, there was only a significant difference in MMP1 expression between the recurrence and non-recurrence groups (*p* = 0.000). In contrast, in the lobular type, there was no significant difference in MMP1 expression between the non-recurrence and recurrence groups (*p* = 0.102) (Table 5).

RETRACTED

**Table 5:** Statistical test results of matrix metalloproteinase (MMP1) expression for ductal and lobular types

Invasive breast cancer type	MMP1 expression		*p*
	Non-recurrence	Recurrence	
Ductal	1.48 ± 1.13	3.24 ± 1.77	0.000*
	1.20 (0.3–4.6)	3.00 (1.1–7.3)	
Lobular	9.43 ± 9.31	17.76 ± 7.56	0.102**
	7.65 (0.0–21.2)	19.80 (6.9–28.5)	
p	0.211*	0.002**	

* Mann-Whitney test

** Independent t-test

Table 5 Matrix metalloproteinase (MMP1) expression test results for ductal and lobular types.

According to the α-SMA expression results, there was no significant difference (*p* = 0.063) in the lobular type and a significant difference (*p* = 0.000) in the ductal type (Table 6).

**Table 6:** Statistical test results of expression α-SMA for ductal and lobular types

Invasive breast cancer type	α-SMA expression		*p*
	Non-recurrence	Recurrence	
Ductal	3.08 ± 1.37	5.59 ± 1.85	0.000*
	3.00 (0.4–5.4)	5.10 (3.2–12.8)	
Lobular	10.12 ± 6.40	22.13 ± 9.39	0.063*
	13.70 (0.0–15.0)	23.90 (9.9–31.5)	
p	0.030*	0.000*	

The Mann-Whitney test *

Table 6 Results of the α-SMA statistical test for ductal and lobular types.

Based on the test results, there was a significant difference in CD95 expression for both cancer types (*p* = 0.000 for the ductal type and *p* = 0.045 for the lobular type) between the groups that experienced recurrence and those that did not (Table 7).

**Table 7:** Statistical test results of CD95 expression for ductal and lobular types

Invasive breast cancer type	CD95 expression		*p*
	Non-recurrence	Recurrence	
Ductal	8.22 ± 5.92	0.92 ± 0.78	0.000*
	6.20 (0.4–5.4)	0.60 (0.0–2.7)	
Lobular	13.17 ± 6.80	1.53 ± 0.69	0.045*
	14.90 (0.0–18.7)	1.80 (0.4–2.4)	
p	0.140*	0.064*	

Mann-Whitney test

Table 6 Results of the α-SMA statistical test for ductal and lobular types.

Based on the test results, there was a significant difference in CD95 expression for both cancer types (p = 0.000 for the ductal type and p = 0.045 for the lobular type) between the groups that experienced recurrence and those that did not (Table 7).

#### Analysis of pathways

A pathway analysis was performed to examine the mechanism of recurrence. Figure 1 shows the findings of the pathway analysis for ductal breast cancer, and Fig. 2 show the results for the lobular type.

**Fig. 1:** Findings from adjuvant chemotherapy and recurrence mechanism pathway study in ductal type breast cancer after mastectomy. A solid arrow indicates a correlation; a dotted arrow indicates none

**Fig. 2:** Results of adjuvant treatment and recurrence mechanism pathway analysis in lobular type breast cancer following mastectomy. A solid arrow indicates a correlation; a dotted arrow indicates none

These findings led to the discovery that, in contrast to lobular-type breast cancer, the recurrence mechanism in early stage ductal-type breast cancer following mastectomy and chemotherapy is distinct. The recurrence mechanism in ductal-type cancer cells occurs through two pathways: the α-SMA pathway, which changes the extracellular structure of cancer cells, and the CD95 pathway, which suppresses the immune response. The CD95 pathway was the only known recurrence mechanism for the lobular type in this study. The lobular type of recurrence process can explain why it is unclear in the lobular type if alterations in the extracellular matrix of cancer cells will make it challenging to identify the tumor’s outer boundary.

RETRACTED

## Discussion

### Breast cancer recurrence and the tumor microenvironment

One of the primary causes of tumor growth, metastasis, and chemotherapy resistance is the tumor microenvironment (TME), which has long been the subject of research aimed at identifying the biological characteristics of tumor cells. Numerous studies have noted that there is two-way communication between tumor cells and the TME, which enables tumor cells to evade the body’s defenses, survive chemotherapy, and spread to new locations [1].

Before BCa reaches the invasive stage, at which point it can spread to the rest of the body, it is referred to as a pre-invasive lesion (Fig. 3). In pre-invasive lesions, cancerous cells are confined to the ducts or lobules from which they originate, and have not yet broken the basement membrane [22]. Breast cancer can originate from either the lobular or ductal epithelium, with lobular carcinomas accounting for 4–10% of the diagnoses. Pre-invasive lesions, known as pre-invasive lesions in ductal carcinoma, are categorized as atypical ductal hyperplasia (ADH) or ductal carcinoma in situ (DCIS) [1, 2, 23]. ADH lesions are small irregularly filled ducts with greater proliferation than usual ductal hyperplasia. Women with ADH lesions are four times more likely to develop breast cancer [3].

**Fig. 3:** Stages of breast cancer development. Tumour cell initiation and expansion within the mammary ducts characterises atypical ductal hyperplasia (A. BCa can be categorized as luminal, HER2-positive, basal, or Claudin-low [9–11, 21]

Invasive ductal carcinomas (IDCs) are tumors that have penetrated the basement membrane and spread over the surrounding stroma, no longer restricted to the impacted duct [22]. The invasive tumors can be classified into different subtypes based on the presence of growth factor or hormone receptors. These consist of triple negative (TNBC) BCa, human epidermal growth factor receptor 2 (HER2)-positive, and estrogen receptor-positive (ER+) BCa [10]. Neither growth factor nor hormone receptors are expressed by TNBC. Moreover, BCa can be categorized as either HER2+ (which expresses amplification of the human epidermal growth factor receptor 2 (HER2) gene but is negative for ER) or luminal (which might be ER+, ER−, or ER + HER2+) based on molecular features. Lastly, there are two kinds known as Basal and Claudin low that are devoid of any growth factors [11]. See Fig. 3.

RETRACTED

### The immune system and cancer

In addition to uncontrolled cell proliferation and escape from apoptosis, cancer cells have immune-manipulating pathways [12]. Tumors can alter their immune microenvironment by signaling immunosuppression, evading immune identification, or increasing inflammation to advance their malignancy. Mutated cells can activate leukocytes to promote malignant tumor cell transformation [12].

This suggests the possibility of cancer immunoediting. The immune system protects and stimulate tumors [13]. Cancer immunoediting includes three phases: elimination, equilibrium, and escape (Fig. 2) [24]. The innate and adaptive immune systems initially recognize tumor-specific antigens, which then results in inflammation [24]. The cancer immunosurveillance network works together to kill tumor cells, limiting further growth. Tumors reach equilibrium only if immunosurveillance fails. Cancerous cells in harmony with their surroundings are more likely to mutate and form novel tumor variants [24]. Tumor cells can use immunosuppressive pathways to escape the immune system during their final stages [24]. These immunologically shaped tumors develop under less selective pressure, produce an immunosuppressive milieu, and are clinically visible. See Fig. 4.

**Fig. 4:** The three phases of cancer immunoediting. Normal cells transition to tumour cells expressing specific tumour antigens, calreticulin, and NKG2D ligands if subject to oncogenic mutational transformation

There are three immunoediting steps in cancer treatment. Oncogenic mutations transform normal cells into tumor cells with tumor antigens, calreticulin, and NKG2D ligands. Cancer immunoediting begins with elimination, where innate and adaptive immune cells assault tumor cells by secreting cytokines, such as IFNγ, IFNα, IFNβ, IL-12, and TNF. In the second phase, equilibrium and selection pressures create new genetic variants in tumor cells. These genetic alterations allow tumors to evade the immune system and enter the third phase of escape, where they develop and become palpable. Immune evasion is influenced by factors such as tumor cell PD-L1 upregulation, cytokine secretion (IL-6, IL-10, TGFβ, and MCSF), and immune cell recruitment (M2 macrophages, TReg cells, and MDSCs) that inhibit NK and CD8+ T cell killing. Downregulation of tumor antigens, calreticulin, and NKG2D ligands reduces the immunological detection of cancer cells [14].

RETRACTED

### The adaptive immune system

The immune system, which comprises innate and adaptive immunity, protects against various microorganisms, infections, and illnesses. Its dynamic network targets infections, establishes immunological memory, and is crucial for BCa formation and progression [15].

### TILs and BCa

TILs, which are immune cells infiltrating cancer tissue, are associated with favorable prognosis and treatment response in TNBC and HER2+ illnesses. In ER+ illnesses, basic TIL numbers are unreliable. TILs predict higher pathological complete responses to neoadjuvant treatment [16–20, 25]. The International TILs Working Group focuses on stromal TILs in H&E-stained tumor sections. Standards and tutorials exist for measuring TILs in invasive tumors, metastases, and DCIS lesions [26, 27].

### Immune regulation in invasive BCa

Initial invasive tumors contain more TILs, with T cells, particularly CD8+ cytotoxic T lymphocytes, dominating the TIL population in breast cancer. TRM cells display immunological checkpoint molecules that help eliminate tumors and are implicated in BCa immunosurveillance. T helper cells, which are type 1 (Th1) polarized and release cytokines, inhibit the immune system and contribute to the pro-tumor immune response, resulting in poor prognosis for breast carcinomas [18–20, 25–31].

In addition to T cells, macrophages, NK cells, and dendritic cells (DCs) infiltrate breast tumors and inhibit tumor growth while promoting tumor growth. The immune system can promote and suppress tumors through various subsets including CD8+, CD4+, TRM, B, NK, M1 macrophages, and dendritic cells. TAM macrophages infiltrate tumors and worsen prognosis in several malignancies [17, 18, 20].

MDSCs are progenitor and immature myeloid-lineage cells that inhibit immune system activation, and high MDSC levels are associated with a poor prognosis. DCs can deliver antigenic peptides to CD4+ T lymphocytes via MHC Class II, activating tumor-specific effector T lymphocytes to attack the tumor and shape the host response to malignant cells [16–20, 25–28].

NK cells have innate and adaptive immunological characteristics and produce pro-inflammatory cytokines that attract and stimulate other immune cells to fight cancer. B lymphocytes are CD20+ adaptive immune cells that produce and secrete immunoglobulin-based antibodies that recognize tumor antigens to provide humoral immunity. B cells help T cells fight by presenting antigens and co-stimulatory chemicals, leading to a regulatory phenotype in B cells, TGF-β production, and CD4+ T cell transformation into immunosuppressive regulatory cells [18, 19, 31, 32].

RETRACTED

In addition to T cells, macrophages, NK cells, and dendritic cells (DCs) also infiltrate breast tumors (Fig. 3) [14, 32, 33]. CD4+ T helper cells, CD8+ CTLs, NK cells, M1 macrophages, and DCs inhibit tumor growth [34]. Conversely, CD4+ FOXP3+ Th2 cells, M2 macrophages, and MDSCs promote tumor growth [34]. See fig. 5.

**Fig. 5:** The immune microenvironment of invasive ductal carcinoma. Subsets of the immune system can elicit both tumour-promoting and tumour-suppressing effects

Fibroblasts, which are not immune cells, create extracellular matrix (ECM) proteins, such as collagen, in the breast stromal milieu and work with stromal microenvironmental immune cells by producing and responding to cytokines [9–13]. CAFs promote tumor growth more than normal fibroblasts do and release pro-inflammatory cytokines, influencing tumor cell EMT and chronic inflammation in the tumor microenvironment [12–15, 24].

### DCIS immune regulation

The pre-invasive stage of breast cancer (BCa) shows significant immune infiltration, with higher T, B, and macrophage levels in DCIS than in normal breasts. Women with DCIS have higher neutrophil levels and more CD4+ T cells, CD20+ B cells, and CD68+ macrophages. CAFs may help DCIS to become IDC by secreting substances that alter the stromal matrix. Recurrent DCIS is defined as the recurrence of DCIS lesions after diagnosis, treatment, or progression to an invasive disease. Patients with low T cell counts and abundant macrophages had the highest DCIS recurrence risk. DCIS has a stronger inflammatory response to malignant cells and more activated effector cytotoxic T cells than IDC do. Exhaustion occurs when CD8+ T cells lose function and express more co-inhibitory receptors after persistent infection [15–20, 25–62].

Retrospective studies of preserved human tumours have demonstrated that M2 macrophages are significantly associated with poor prognosis in both ER- and ER+ tumours [16].

### Immune control of hyperplasia

Early hyperplastic breast tumorigenesis is less well-characterized than DCIS, with limited data on breast ADH immune infiltrates. DCIS with a greater fraction of genome alterations had more TILs, suggesting that genetic alterations may activate the immune system early. Immune engagement increases hyperplastic tissue proliferation, with early malignancies and tumorigenesis linked to macrophage numbers and inflammatory cytokines. Normal breast tissue from women with high breast density contains more macrophages, DCs, B cells, and CD4+ T cells, suggesting pro-tumor Th2 polarization [20, 25, 26]. Limited information on hyperplastic lesions may be related to their modest size and close association with low-grade DCIS. Fibroblasts may also help initiate tumor growth, with research suggesting that stromal-specific TGFβ-RII inactivation causes pre-invasive prostate cancer lesions in mice and loss of PTEN can promote BCa growth. Immunotherapies, such as those targeting the anti-PD-1/PD-L1 inhibitory pathway, have shown promise as innovative treatments for TNBC and HER2+ cancer. Innate immunity, an alternative immune-based therapy, is also being explored, with novel therapies such as anti-CSF1R blocking TAMs’ receptors that recruit and activate M2 pro-tumor immune cells [27–33, 35].

RETRACTED

### Immune-based BCa growth and progression treatments

Elevated stromal lymphocyte counts in IDC and DCIS are prognostic indicators for TNBC and HER2+ cancers. Immunotherapies, specifically those targeting the PD-1/PD-L1 inhibitory pathway, can mobilize the immune system against BCa. Anti-PD-L1 therapy is promising for TNBC and DCIS because it reduces tumor volume and increases immunogenicity. Trials have examined this therapy alone or in combination with HER2-specific treatments [34, 36–48].

Mesenchymal markers such as vimentin, N-cadherin, and fibronectin can be used to detect epithelial-to-mesenchymal transition (EMT), which is a key factor in the process of recurrence and the emergence of chemotherapeutic drug resistance. The primary constituent of the cytoskeleton or cell skeleton is vitreolin. Moreover, vimentin participates in cell movement and forms the cellular skeleton. Actively dividing cells express vitreolins. Higher expression of vimentin has been linked to more aggressive characteristics of tumor cells, an increased capacity for metastasis, and worse prognosis [29–31]. The actin structure of the cytoskeleton is an essential component in protrusion and cell migration, indicating that the intermediate cytoskeleton filament, particularly vimentin, also contributes to adhesion and cell spread [31, 35]. Vimentin can also protect cells from stress.

Certain forms of cancer, such as primary epithelial carcinoma or metastases, exhibit abnormal expression of vimentin. According to recent research, vimentin also contributes to the EMT process in breast cancer, reducing the expression of genes linked to invasion and similar basal phenotypes [32]. Patients with breast cancer expressing high levels of this substance have a poor prognosis. Furthermore, studies conducted in 2013 by Cairo University in 2021 revealed a significant correlation between high levels of vimentin and poor prognosis for recurrent breast cancer [36]. Vimentin activation of the AKT pathway is linked to the increased proliferation and invasion of breast cancer cells [37]. High levels of vimentin are also significantly associated with the spread and survival of breast cancer cells, allowing for cancer recurrence.

RETRACTED

Statistical tests revealed significant variations in vimentin expression between the ductal type (*p* = 0.000) and lobular type (*p* = 0.021) groups that experienced recurrence events and those that did not. Research by Vora in 2009 also produced similar results, namely recurrent breast cancer patients with higher vimentin levels compared to non-recurrent breast cancer, both in lobular and ductal breast cancer types [37, 40]. A study by Rodrigez stated that vimentin expression in non-basal-like tumors was lower than that in basal-like tumors (i.e., patients with recurrent breast cancer). This result is consistent with the findings of Wang (2020), who reported vimentin overexpression in ductal-type breast cancer cells [38]. This is due to the synergy between vimentin and LAP3, where LAP3 expression can increase vimentin expression [38]. In addition, the relationship between the two can be significant. Vimentin expression in tumor cells corresponds with recurrence, and basal-like tumors are associated with poor prognosis and a tendency to recur [41]. However, Seshadri’s 1996 study produced different results. According to this study, there was no meaningful correlation between vimentin expression and the chance of dying or recurrence of breast cancer. The authors of the same study also clarified that vimentin is only important in cancers with negative hormone receptors [42].

In our investigation, there was no significant difference in MMP1 expression between the lobular type (*p* = 0.102), but there was a significant difference in MMP1 expression for the ductal type between the recurrence and non-recurrence groups (p = 0.000). A study by Del Caszar et al. found that increased MMP1 expression is more common in ductal-type breast cancer than in lobular and mucinous types [43]. Shen et al. also found that increased MMP1 expression in invasive breast cancer is linked to multidrug resistance, which is resistant to chemotherapy drugs [44]. In addition to chemoresistance, increased MMP1 expression has been linked to resistance to hormonal therapy [45].. Another study found that increased MMP1 expression in breast cancer was correlated with metastasis and recurrence, suggesting that MMP1 can be used as a prognostic factor in breast cancer [46].

Cancer cells use the TGF pathway to stimulate increased PDGF expression during the EMT phase of breast cancer. TGF-β regulates homeostasis in healthy cells, upholds the body’s defense mechanisms, and aids in wound healing. TGF-β inhibits tumor growth in premalignant cells either directly (by activating apoptosis, for example) or indirectly (by regulating the stroma surrounding the cells, such as by reducing inflammation). The capacity of TGF-β to inhibit tumor growth can be deactivated by malignant cells after EMT has taken place, making its role as a trigger for tumor advancement the dominant function [47].

RETRACTED

After undergoing epithelial-mesenchymal transition, cancer cells use TGF-β to trigger the production of pro-tumorigenic cytokines such as platelet-derived growth factor (PDGF), hepatocyte growth factor (HGF), ILEI (interleukin-like EMT-inducer), and epidermal growth factor) [48]. PDGF is a pro-angiogenic factor that participates in both autocrine and paracrine processes during the growth of solid tumors. The PDGF signal makes the tumor cells more autocrine (aggressive) and paracrine (helps blood vessels grow). It also transforms healthy fibroblasts into cancer-associated fibroblasts (CAF). Moreover, CAF activate transcription factors that can change epithelial progenitor cells into mesenchymal progenitor cells, including SNAIL and SLUG. More cells undergo EMT as a result of these processes, and “loop signaling” enables cancer cells to proliferate and spread [49].

CAFs are the most prevalent element in the tumor microenvironment is CAF. When a tumor is malignant, CAF control its growth by controlling its nutrition, reshaping the extracellular matrix to facilitate cancer cell invasion, suppressing the immune system to prevent immune cells from killing cancer cells, and controlling extra- and intracellular signals to allow cancer cells to withstand chemotherapy [23]. CAF have multiple markers, including α-SMA, FAP, and integrin β1/CD29, of which α-SMA is the most commonly used [51].

In this study, PDGF expression in the ductal type (*p* = 0.000) and lobular groups (*p* = 0.002) showed significant differences between the recurrence and non-recurrence groups. These findings are consistent with those of Jansson, who found that PDGF expression is linked to the incidence of early recurrence in breast cancer [52]. Another study by Chou found that breast cancer patients receiving taxane chemotherapy may develop chemoresistance if their PDGF expression is overexpressed [53]. Another study found that inhibiting PDGF expression in patients with breast cancer improved the efficacy of hormonal therapy in patients who tested positive for hormonal receptors [54].

The expression of α-SMA revealed a significant difference (p = 0.000) between the non-recurrence and recurrence groups for ductal-type breast cancer. These findings align with Bonneau’s research, which found that in luminal (ductal)-type breast cancer, α-SMA (CAF) expression correlates with metastasis and recurrence [55, 56]. In lobular breast cancer, α-SMA expression did not differ significantly between the recurrence and non-recurrence groups (*p* = 0.063). These findings were obtained because, in contrast to ductal-type breast cancer, lobular-type breast cancer does not exhibit severe TME changes [43]. Recurrence in lobular-type breast cancer is frequently the result of a non-radical margin of operation because the tumor’s outer boundary is difficult for pathologists and surgeons to determine owing to unclear TME changes.

RETRACTED

### Recurrence of breast cancer: immunity escape

Any breast cancer cells that remained latent after treatment (chemotherapy, radiation, or surgery) were removed. In a latent state, cancer cells try to withstand chemotherapy and radiation, adapt to new microenvironments, and defend the body’s defense mechanisms [57].

When breast cancer cells transition from an epithelial to a mesenchymal phenotype (EMT), it is a crucial stage in their development to emerge from a dormant state. For cancer cells to become immortal and possess characteristics of cancer stem cells, the EMT process causes the cells to change pro-apoptotic factors into non-apoptotic ones. If cancer cells are already in this state, they will be more aggressive, more resistant to multidrug chemotherapy, and more likely to return [58].

CD95 is a pro-apoptotic factor crucial for regulating the proliferation of cancer cells. The death-inducing signaling complex (DISC) is activated by cancer cells viaough the Fas-associated protein with death domain (FADD), caspase-8, and caspase-10 pathways. 60 CD95 can change from a pro-apoptotic factor to a non-apoptotic factor when EMT occurs or when it is continuously stimulated. 61 IFNα or IFN^2^ are released by cancer cells when they undergo EMT or long-term stimulation of CD95. These proteins interact with IFNAR1 and IFNAR2 to induce cell death. This connection results in STAT1-promoting cancer stemness by activating signal transducer and activator of transcription 1 (STAT1) [61].

The study findings demonstrated a significant difference in CD95 expression in the lobular type (*p* = 0.045) and ductal type (*p* = 0.000) between the groups that had recurrences and those that did not. Pellegrino reported similar findings, stating that CD95 expression is a risk factor for breast cancer recurrence [59].

Mechanisms of recurrence in breast cancer of the ductal and lobular types.

RETRACTED

Mechanisms of local recurrence in breast cancer of the ductal type.

The findings of the pathway analysis in ductal type recurrence breast cancer in this study demonstrated a strong association (β = 0.611) and a substantial influence between vimentin and MMP1 expression (*p* = 0.000). These findings are consistent with studies on Rac1b cells by Stallings-Mann (2012), who demonstrated that vimentin increases MMP1 expression [55–58].

Additionally, there was a significant correlation (β = 0.670) between vitretin and PDGF expression (*p* = 0.000). This result is consistent with that of Paulin (2022), who found that binding of basic protein heterodimers, leucine-zipper (bZIP), Jun (c-Jun, JunB, JunD), Fos (cFos, FosB, Fra1, and Fra2), ATF (ATF-1, ATF-2)/CREB, or homodimers from Jun/Jun, affects several growth factors, including PDGF [58].

In this study, PDGF also had a somewhat correlated (β = 0.592), but a significant effect on α-SMA expression (*p* = 0.000). Similar findings were also found in a 1998 study. The study also mentioned that vimentin is reorganized when the PDGF receptor is activated, and this process is linked to fibroblast cancer, in which α-SMA is a marker [59].

In this study, there was a moderate correlation (β = 0.592) between α-SMA expression and the incidence of recurrence in ductal-type breast cancer (*p* = 0.000). These data are consistent with those of a study by Bonneau that found CAF to be correlated with the incidence of recurrence in early stage ductal-type breast cancer [55]. Another study by Risom found that CAF activation alters the structure and composition of the cancer cell stroma, making it more aggressive and increasing the risk of recurrence [62].

EMT, which weakens the body’s defenses, also affected the recurrence rate in this study. In this study, pathway analysis revealed that EMT had a moderate association (β = 0.592) with a *p*-value of 0.000 for CD95 impact. Moreover, there was a strong correlation (*P* = 0.000) between CD95 expression and the likelihood of recurrence. Guégan also reported this in a prior study, noting that in ductal-type breast cancer, CD95 expression was associated with resistance to chemotherapy and recurrence [60].

Mechanisms of local recurrence in breast cancer of the lobular type.

In this study, the inability of the body’s defense system to eliminate cancer cells affected the recurrence of lobular-type breast cancer. In this trial, TME had no discernible impact on the likelihood of recurrence. Van der Sangen’s research revealed that TME in the case of lobular-type breast cancer influences the likelihood of recurrence in the event that less drastic surgery is performed [59].

CD95 showed a moderate correlation coefficient (β = 0.467) and was a significant non-apoptotic factor (p = 0.000) in lobular breast cancer owing to the EMT process. These alterations endow cancer cells with immortality and characteristics similar to cancer stem cells [61]. This study demonstrated that CD95 influences the likelihood of recurrence (*p* = 0.001) and exhibits a substantial connection (β = 0.802). The immortality of cancer cells renders them resistant to chemotherapy, which increases their risk of recurrence. These findings are consistent with a study by Wilson, who found that, in contrast to ductal-type breast cancer, lobular-type breast cancer is more resistant to chemotherapy [54–62].

RETRACTED

The number of cells expressing vimentin, MMP1, and PDGF in ductal-type tumors was shown to be different from that in lobular-type cases that experienced local recurrence following mastectomy and adjuvant chemotherapy, based on the findings of observations and statistical analysis. Conversely, we did not observe any variation in α-SMA or CD95 expression. In addition, the ductal form of early stage breast cancer has a different local recurrence mechanism than the lobular type [63]. The ductal form of cancer has a recurrence mechanism that involves two pathways: one that impacts the tumor microenvironment, and the other that targets the body’s defense mechanisms. In contrast, the only pathways that can cause the local recurrence of lobular breast cancer are those that affect the body’s defense mechanisms. The author acknowledges the high degree of heterogeneity in breast cancer cases and points out that the limitations of the study were the limited sample size and heterogeneity. Further research involving many centers may prove to be beneficial.

### In summary

While the tumor microenvironment and immune system both have an impact on the recurrence of IDC, the immune system is more important in ILC. This study suggests that enhancing the immune system may be an effective cancer treatment.

BCa tumors have an immune microenvironment, with invasive lesions primarily containing T lymphocytes, particularly CD8+ CTLs. Invasive lesions may be influenced by cytokines at the cancer site, whereas stromal microenvironments may contain both innate and adaptive cells. Pre-invasive BCa stages, such as DCIS and ADH, may have low T cell counts and high macrophage counts. Genetic abnormalities in ADH lesions may activate the immune system.

## Data Availability

A database is available to the corresponding author. The database is available upon review and request. All authors have shared the database.
